The article "A Multicentre Randomized Controlled Clinical Study of Cross Electro-Nape-Acupuncture (CENA) for the Treatment of Pseudobulbar Palsy in Patients with Tracheotomy Intubation for Severe Cerebral Haemorrhage" was retracted in 2023. Reasons: signs of a paper mill; compromised peer review; unreliable results or conclusions.

# A Multicentre Randomized Controlled Clinical Study of Cross Electro-Nape-Acupuncture (CENA) for the Treatment of Pseudobulbar Palsy in Patients with Tracheotomy Intubation for Severe Cerebral Haemorrhage

**DOI:** 10.1155/2023/9304934

**Published:** 2023-04-27

**Authors:** Shengnan Xu, Sihui Guo, Manchao Sun, Cheng Cui, Ke Xu, Xue He, Yanan Cui, Ziyin Gao, Zhenqi Wu, Jiaxin Xue, Yucai Ma, Jiahong Sun, Rui Zhang, Guoliang Cai, Guofeng Cai

**Affiliations:** ^1^Heilongjiang University of Traditional Chinese Medicine, Harbin, China; ^2^Postdoctoral Research Workstation of Skiing Teaching and Training Base of Harbin Sport University, 150008 Harbin, China; ^3^College of Sports and Human Sciences, Harbin Sport University, 150008 Harbin, China

## Abstract

**Objective:**

The objective is to evaluate the clinical efficacy of cross electro-nape-acupuncture (CENA) in the treatment of pseudobulbar palsy in patients with tracheotomy intubation for severe cerebral haemorrhage and to provide an innovative acupuncture method for the treatment of such patients.

**Methods:**

A total of 126 patients from six trial centres who met the inclusion criteria were randomly divided into three groups according to the random number table method in the ratio of 1 : 1 : 1, with 42 patients in each group, and the three groups were divided into CENA group, electro-acupuncture group, and acupuncture group. Each group's acupuncture treatment lasted for 30 minutes, and the needles were removed at the end of the treatment. Acupuncture was performed once a week on Sunday only and twice a day from Monday to Saturday, a total of 4 weeks of treatment. The SWT, FDA, ChSWAL-QOL, and TCRGS scores of the three groups of patients before and after treatment were compared to evaluate the effect of CENA on remodelling the function of swallowing reflex and cough reflex and promoting the recovery of dysarthria and swallowing quality of life in pseudobulbar palsy in patients with tracheotomy intubation for severe cerebral haemorrhage.

**Results:**

After treatment, the WST and TCRGS grade scores decreased and the FDA and ChSWAL-QOL scores increased significantly in all three groups compared with the pretreatment scores and were statistically significant. There was a significant difference between the three groups for these four indicators after treatment; the comparison between groups showed significant differences in the CENA group compared to the electro-acupuncture and acupuncture groups. The efficiency of the CENA group was significantly better than that of the electro-acupuncture and acupuncture groups.

**Conclusion:**

Compared with the acupuncture and electro-acupuncture groups, the CENA could better promote the remodelling of swallowing function and cough reflex function, promote the recovery of dysarthria, and better improve the quality of life of patients with pseudobulbar palsy from tracheotomy intubation in severe cerebral haemorrhage.

## 1. Introduction

Haemorrhage of more than 30 ml above the cerebellar curtain is called severe cerebral haemorrhage, and respiratory failure and pseudobulbar palsy are serious complications that accompany severe cerebral haemorrhage [1]. Cerebral haemorrhage occurs when a blood vessel in the brain ruptures and blood flows out at the rupture and is associated with a variety of cardiovascular and cerebrovascular disease factors, thus most patients with cerebral haemorrhage are accompanied by hypertension [2]. Many factors can increase the risk of cerebral haemorrhage, most notably poor lifestyle habits and complications from other clinical conditions [3]. Due to the compression of the respiratory centre of the brainstem after haemorrhage, significant oedema of the brain tissue, and the formation of hypostatic pneumonia after prolonged bed rest, the patient's respiratory failure was improved by tracheotomy intubation and ventilator-assisted ventilation when the patient was in respiratory failure [4, 5].

Pseudomyelination palsy is an upper motor injury caused by bilateral interference with the cortical medullary tracts [6]. The corticomedullary tract exerts supranuclear control over the motor nuclei of the brainstem and is involved in muscle movements of the head and neck, which originate from pyramidal cells in the cortex and terminate in the cranial nerve nuclei that control mastication, swallowing, and speech [7]. Pseudomyelination is characterized by dysarthria, dysphagia, facial and tongue weakness, and emotional instability, so any condition that damages the cortical medullary pathways bilaterally can lead to pseudomyelination [8]. Swallowing impairment can directly affect feeding and nutrient absorption, with most patients being fed nasally, which is very painful, and is rejected by the patient due to inability to express themselves because of speech impairment, as well as increasing the likelihood of aspiration pneumonia due to swallowing impairment and aspiration, exacerbating lung infections and impairing recovery of respiratory function [9]. The presence of a foreign body in the airway (tracheotomy tube) also hinders the patient's recovery of swallowing function. This creates a vicious circle that can be life threatening [10]. Therefore, we need effective treatment to fully restore swallowing and respiratory function.

Crossed electro-neck-acupuncture (CENA) works by regulating the balance of the body and has the effect of enhancing metabolism [11]. Electro-acupuncture is a method of preventing and treating disease by inserting a millineedle into acupuncture points to obtain true qi, and then applying the pulse current output from the electro-acupuncture instrument to the meridians and acupuncture points in the body through the millineedle, which has good electrophysiological properties [12]. It regulates and balances the meridians and organs of acupuncture points, promotes blood circulation, boosts metabolism, reduces inflammation and pain, and restores normal function to tissues and organs in a pathological state [13]. Electroacupuncture is more stimulating and more effective than traditional acupuncture, but in patients with spasticity, electro-acupuncture can stimulate the muscles leading to increased spasticity, whereas traditional acupuncture can adjust the technique to avoid aggravating the symptoms [14].

This trial evaluated the clinical efficacy of CENA for the treatment of pseudobulbar palsy with tracheotomy intubation in severe cerebral haemorrhage in order to provide an innovative acupuncture approach for the treatment of such patients.

## 2. Materials and Methods

### 2.1. General Information

#### 2.1.1. Baseline Data

A total of 126 patients from six trial centres:

1. The Second Hospital of Heilongjiang University of Traditional Chinese Medicine, Hanan Branch
2. The Second Hospital of Heilongjiang University of Traditional Chinese Medicine
3. The Second Hospital of Dalian Medical University
4. Xiaotangshan Hospital, Beijing
5. Shenzhen Longhua District Central Hospital
6. Yulin Central Hospital, Shaanxi Province) were admitted to this pilot study, and the hospitalization period was from November 2021 to March 2022

#### 2.1.2. Randomization and Blinding

*(1) Grouping Methods*. The 126 trial study subjects who met the diagnostic criteria and agreed to be enrolled were randomly divided into three groups in the order of consultation using the random number table method in the ratio of 1 : 1 : 1, with 42 patients in each group, and the three groups were divided into the CENA group, the electro-acupuncture group, and the acupuncture group. A random assignment card was prepared, which included serial number, group, random number, and treatment method. The random assignment cards were again kept by dedicated personnel, and when qualified subjects entered the study, the envelopes with the same serial numbers were opened in the order of their entry, and treatment was given according to the groups specified in their cards, and 21 patients in each of the six clinical centres.

*(2) Evaluation Methods*. The blinded evaluation was used during the study, with separation of implementer, recorder, and evaluator. The trial followed the Declaration of Helsinki, and the study was approved by the Ethics Committee of the Second Hospital of Heilongjiang University of Traditional Chinese Medicine (acceptance number 2022-K44).

### 2.2. Criteria

#### 2.2.1. Diagnostic Criteria

1. Diagnostic criteria for severe cerebral haemorrhage refer to the “Chinese Consensus on the Management of Severe Cerebrovascular Disease 2015” [1]: The determination of severe cerebral haemorrhage is based on the size of intracranial haematoma, which can be defined as severe cerebral haemorrhage when the size of haematoma is more than 30 ml (supratentorial cerebellar) in clinical patients.
2. Diagnostic criteria for pseudobulbar palsy refer to “Neurological Disease Syndromes [15]”: ① Speech difficulty, vocal difficulty, and feeding difficulty; ② positive pathological brainstem reflexes, such as sucking reflex and palmar chin reflex; ③ emotional disorders, such as strong crying and laughing; and ④ loss of soft palate reflex and weak or normal pharyngeal reflex.

The diagnosis can be confirmed if any one of the above ① and ②∼④ is met.

#### 2.2.2. Inclusion Criteria

1. The location of the patient's lesion was confirmed by cranial CT or cranial MRI examination to be below the cerebral cortex and above the brainstem region.
2. Patients met the diagnostic criteria for severe cerebral haemorrhage as well as pseudobulbar palsy.
3. Patients aged 18 to 70 years old (including 18 and 70 years old).
4. Patients with swallowing disorders confirmed by the screening of the water swallowing test (SWT ≥ level III).
5. Patients with a first episode and tracheotomy intubation, with a disease duration between 14 and 28 days (including 14 and 28 days) and a stable general status, already off ventilator-assisted ventilation.
6. Patients with a clinical pulmonary infection score (CPIS) ≤ 6.
7. Patients with or without impaired consciousness after the onset of the disease and can complete the relevant treatment as instructed.
8. Patients and patients' family members who agree to join this clinical trial study and have high compliance to actively cooperate with the treatment.
9. Patients and patients' family members signed the informed consent form.

#### 2.2.3. Exclusion Criteria

1. Patients who did not meet the diagnostic criteria for severe cerebral haemorrhage as well as pseudobulbar palsy and the inclusion criteria.
2. Patients with brainstem lesions.
3. Patients with age >70 years old or <18 years old.
4. Patients with combined complete motor aphasia and sensory aphasia.
5. Patients with swallowing dysfunction and speech dysfunction due to other causes, such as oesophageal tumour, myasthenia gravis, Green–Barre syndrome, and localized damage to the pharynx.
6. Patients with serious heart, liver, kidney, lung, and other organ diseases and serious diseases of other systems before or after the onset of the disease.
7. Patients with severe consciousness disorders, mental retardation, or other psychiatric symptoms unable to cooperate with treatment, or those who subjectively refuse to cooperate with participation in clinical studies.
8. Those who have adverse reactions to acupuncture as well as electro-acupuncture treatment.

#### 2.2.4. Rejection Criteria

1. Patients who refused to cooperate and had poor compliance after enrolment.
2. Those who did not follow the treatment protocol during the trial and added other therapies on their own.
3. Those whose clinical data collection was incomplete for various reasons.
4. Patients who were transferred to a hospital or died of serious illness due to deterioration during treatment.
5. Those who had serious adverse events, serious comorbidities, and changed the treatment plan during the course of treatment.
6. Patients who abandoned the treatment and insisted on quitting the trial in the course of treatment.

### 2.3. Methods

#### 2.3.1. Basic Treatment and Nursing Methods

Patients in all groups were given western medicine treatment, including anti-inflammatory therapy (adjustment and use of antibiotics based on sputum culture and drug sensitivity test results), sputum chemotherapy, gastric mucosal protection therapy, nutritional neurotherapy, and other individualized treatments such as regulation of blood glucose, blood lipids, and blood pressure. Also, patients in all groups were given standard care of the respiratory tract, quality humidification with a modified venturi heating and humidifying device, and superficial aspiration to reduce airway injury [16]. In addition, attention was paid to the skin condition around the tracheotomy tube to avoid infection, oral hygiene was enhanced, and the patients were turned and tapped on the back in a timely manner to promote the recovery of the original lung volume.

#### 2.3.2. Acupuncture Group

The acupuncture points were selected according to the acupuncture points of stroke disease in Acupuncture and Moxibustion Therapeutics (the first edition of the 12th Five-Year Plan textbook in 2014) [17]; bilateral acupuncture points are taken for treatment, and the specific points are shown in Table 1. Acupuncture treatment was performed after routine disinfection with 75% ethanol, and Huatuo brand needles with a size of 0.35 × 40 mm were utilized. Each acupuncture treatment lasted 30 minutes, and the needles were removed at the end of the treatment. Acupuncture was performed once a week on Sunday only, and twice a day from Monday to Saturday, a total of 4 weeks of treatment.

#### 2.3.3. Electro-Acupuncture Group

The electro-acupuncture group was energized based on the acupuncture group. The KWD-808 pulse acupuncture instrument was used, and the ipsilateral TE17 and GB20 were connected to the electro-acupuncture instrument after the acupuncture was completed. That is, the positive side of the same electrode line is connected to the left TE17, and the negative side is connected to the left GB20, the same for the right side. The wave type of the acupuncture instrument was selected as a continuous wave, the frequency was set at 1.5 Hz, and the current intensity was adjusted by rotating the scale to 6, which could be simply adjusted according to the general state of the patient. The acupuncture time and duration of treatment were the same as the acupuncture group.

#### 2.3.4. Cross Electro-Nape-Acupuncture (CENA) Group

The CENA group was given cross electro-nape-acupuncture on the basis of the acupuncture group. The selection of the acupuncture instrument and the current level was the same as that of the electro-acupuncture group. After the acupuncture is completed, apply the acupuncture treatment instrument to cross the TE17 and GB20 on both sides with electricity, which means, the positive side of one electrode wire was connected to the left TE17, and the negative side was connected to the right GB20. In addition, the positive side of another electrode is connected to the right TE17, and the negative side is connected to the left GB20 (the specific connection can be seen in Figure 1). The acupuncture time and duration of treatment were the same as the acupuncture group and electro-acupuncture group.

### 2.4. Therapeutic Effects

#### 2.4.1. Observation Indicator

*(1) The Water Swallowing Test (WST)*. WST was first proposed by the Japanese scholar Toshio Kubota [18] and is often used in clinical practice to detect aspiration and prevent pneumonia and assess swallowing function. It is a standardized test used worldwide [19], but the amount of water given varies depending on the patients, and we chose to give 30 ml of water for the test. The test levels are detailed in Table 2.

*(2) The Frenchay Dysarthria Assessment (FDA)*. FDA was introduced by Enderby in 1980 [20]. This tool quantitatively assesses speech-related organs and provides a measure of intelligibility [21]. The scale is clinically important for the assessment of dysarthria in patients with bulbar palsy. We used the Chinese version of the FDA to assess patients with 8 major items and 28 minor items, with each minor item divided into *a*, *b*, *c*, *d*, and *e* levels (assessment index: number of “*a*” items/total number of items; assessment level: normal: 28–27/28; mild impairment: 26–18/28; moderate impairment: 17–14/28; severe impairment: 13–7/28; and extremely severe impairment: 6–0/28). We performed vocal tests by sealing the tracheotomy intubation of the pneumonectomy patient on the basis of ensuring that the patient's oxygen saturation was greater than 90.

*(3) Chinese Mandarin version Swallowing Quality of Life (ChSWAL-QOL)*. SWAL-QOL questionnaire was designed as a tool for evaluating the QOL of patients with swallowing disorders from physiological, emotional, and social aspects [22–24]. The SWAL-QOL is widely considered the optimum tool for evaluating QOL in patients with swallowing disorders, and this instrument has been translated into many different languages, we chose the ChSWAL-QOL for assessment [25]. This questionnaire consists of a total of 44 entries consisting of 11 factors that affect swallowing, each with 5 different levels, ranging from poor to good on a scale of 1–5: 1 means very compliant; 2 means relatively compliant; 3 means somewhat compliant; 4 means not very compliant; and 5 means not at all compliant. The lower the score, the worse the swallowing function and the poorer the quality of life.

*(4) Tracheostomy Cough Reflex Grading Score (TCRGS)*. TCRGS has a minimum score of 1 point and a maximum score of 5 points; the lower the score, the better the prognosis, it is used to assess cough reflex function and to provide an indicator for extubation in patients with tracheotomy intubation [26, 27]. Detailed scoring levels are listed in Table 3.

### 2.5. Effect Criteria

Efficacy evaluation according to the change in WST grade before and after treatment: cure: normal swallowing and Paddy's drinking water test rating of 1 level; significant effect: significant improvement in dysphagia, Paddy's drinking water test rating of 2 or more levels higher, and not cured; effective: improvement in dysphagia and Paddy's drinking water test rating of 1 level higher; and ineffective: no improvement in dysphagia and Paddy's drinking water test rating unchanged or lowered.

### 2.6. Statistical Analysis

The data were analysed using SPSS25.0 statistical software, and the measurement data conforming to normal distribution were expressed as mean ± standard deviation ($\bar{x}$ ±s), the skewed data were expressed as *M (p25, p75)*, and the skewed multigroup measurement data were expressed as Kruskal–Wallis. The other multiple-group count data splitting two comparisons required adjustment of the calibration level; *α* = *α*/*k*, where *k* is the number of comparisons, and *α* = 0.05 and *p* < 0.05 indicated that the difference was statistically significant.

## 3. Results

A total of six patients fell off during the study, two patients in the CENA group and two patients in the electro-acupuncture group insisted on terminating treatment after improvement, one patient in the acupuncture group insisted on dropping out of the trial, and one patient changed the treatment plan, while the remaining 120 patients completed the treatment.

### 3.1. Baseline Characteristics

There were no differences among the key baseline characteristics of the three groups (Table 4).

### 3.2. Evaluation of SWT, FDA, TCRGS, and ChSWAL-QOL

#### 3.2.1. SWT Scores

There were significant differences before and after treatment in both groups (CENA group: *z* = 5.47, *p* < 0.001; electro-acupuncture group: *z* = 5.16, *p* < 0.001; and acupuncture group: *z* = 4.65, *p* < 0.001), and a significant difference was found in SWT scores between the three groups after treatment (*h* = 24.65, *p* < 0.001).

#### 3.2.2. FDA Scores

There were significant differences before and after treatment in both groups (CENA group: *z* = 5.52, *p* < 0.001; electro-acupuncture group: *z* = 5.45, *p* < 0.001; acupuncture group: *z* = 5.25, *p* < 0.001), and a significant difference was found in FDA scores between the three groups after treatment (*h* = 32.25, *p* < 0.01).

#### 3.2.3. TCRGS Scores

There were significant differences before and after treatment in both groups (CENA group: *z* = 5.47, *p* < 0.001; electro-acupuncture group: *z* = 5.34, *p* < 0.001; and acupuncture group: *z* = 3.94, *p* < 0.001), and a significant difference was found in FDA scores between the three groups after treatment (*h* = 3.33, *p* < 0.001).

#### 3.2.4. ChSWAL-QOL Scores

There were significant differences before and after treatment in both groups (CENA group: *z* = 5.52, *p* < 0.001; electro-acupuncture group: *z* = 5.53, *p* < 0.001; and acupuncture group: *z* *=* 5.52, *p* < 0.001), and a significant difference was found in FDA scores between the three groups after treatment (*h* = 26.89, *p* < 0.001).

The SWT, FDA, TCRGS, and ChSWAL-QOL results are presented in Table 5 and Figure 2.

### 3.3. Evaluation of Efficacy

The efficiency of the three groups after treatment was statistically significant (*x*^*2*^ = 38.7, *p* < 0.001), and the total efficiency of the CENA group, electro-acupuncture group, and acupuncture group were 95%, 85%, and 65%, respectively. The improvement rate of the CENA group was higher than that of the electro-acupuncture group (*x*^*2*^ = 13.16, *p*=0.004) and the acupuncture group (*x*^*2*^ = 37.48, *p* < 0.001) (Table 6 and Figure 3).

### 3.4. Adverse Events

Throughout the experiment, there were no abnormal changes in vital signs or experimental factors in any of the three groups of patients. There were no reports of any serious adverse reactions, such as fainting and broken needles during acupuncture. There were 2, 1, and 2 patients with postacupuncture haematomas in the CENA group, electro-acupuncture group, and acupuncture group, respectively, and these haematomas disappeared after 2 days without any treatment.

## 4. Discussion

With the improvement of living standards and the multiplication of individual stress in today's society, high oil and salt intake, irregular dietary habits, irregular intake of alcohol and tobacco, and irregular living habits have led to an increased incidence of cerebrovascular disease in the modern population, with patients gradually becoming younger [28, 29]. A severe cerebral haemorrhage is defined when the size of the haematoma above the cerebellar curtain exceeds 30 ml [1]. After onset, patients require early tracheotomy intubation for assisted ventilation due to respiratory failure. Patients with combined pseudomyelitis increase the likelihood of aspiration pneumonia due to the presence of foreign bodies in the airway, which exacerbates swallowing disorders and therefore requires the promotion of both the cough reflex and swallowing reflex reconfiguration. Restoration of pulmonary function and early removal of the tracheotomy cannula will also help recovery from pseudobulbar palsy.

Cross electro-nape-acupuncture is a combination of traditional acupuncture and modern medical technology that allows the electric field to act on the cough reflex and swallowing reflex centres in the brainstem, which in turn facilitates the remodelling of the cough reflex (tracheal sealing), the restoration of the swallowing reflex (removal of the gastric tube and transoral feeding), and the restoration of consciousness through complex neural reflex regulation [11–13]. Compared with surgery, the treatment of pseudobulbar palsy by acupuncture is simple, inexpensive, and clinically effective, and is widely used in clinical treatment [30, 31]. As a combination of acupuncture and modern medical techniques, CENA highlights its superior therapeutic effects over traditional acupuncture. Previous studies have shown that CENA not only promotes cough reflex function and swallowing function remodelling in stroke patients but also controls lung infection, accelerates ventilator withdrawal, and promotes recovery from impaired consciousness [32–35]. Therefore, the same CENA method was used in this study to observe its therapeutic effect on patients with severe cerebral haemorrhage tracheotomy intubation with pseudobulbar palsy.

The aim of our study was to observe the therapeutic effect of CENA in the treatment of pseudobulbar palsy in patients with tracheotomy intubation for severe cerebral haemorrhage. After treatment, the WST and TCRGS grade scores decreased and the FDA and SWAL-QOL scores increased significantly in all three groups compared with pretreatment and were statistically significant. Besides, there was a significant difference between the three groups for these four indicators. The difference showed that the CENA group was better than the electro-acupuncture group and the acupuncture group in reducing the WST and TCRGS scores, indicating that CENA was better in restoring the swallowing function and cough reflex function of the patients. The CENA group improved the FDA and SWAL-QOL score better than the electro-acupuncture group and the acupuncture group, indicating that the CENA could better promote the recovery of dysarthria and improve the quality of life of the patients. The efficiency of the CENA group was significantly better than that of the electro-acupuncture and acupuncture groups, The treatment effect of CENA was superior to that of the electro-acupuncture and acupuncture groups.

The effective mechanism of CENA may be related to our choice of acupuncture points and our treatment philosophy, where the efficacy of two acupuncture points, TE17 and GB20, in treating pseudobulbar palsy has been well documented [36, 37]. Due to their specific location, it is important to pay attention to their angle and depth when treating them [38, 39]. In traditional medicine, TE17 is used to treat not only psychiatric disorders such as epilepsy and spasticity but also local disorders of the eyes, ears, face, and mouth, as well as voice loss, and there is a rich neural network running under TE17 [38–40]. GB20 treats a wide range of diseases, mainly caused by various “wind evils,” not only for head, face, ears, eyes, waist, and back diseases, but also for stroke, malaria, schizophrenia, manic-depressive, and other mental illnesses, and the deepest part of the GB20 has the medulla oblongata [39–41]. The horizontal section connecting the bilateral TE17 and GB20 is closest to the brainstem. Based on the properties of direct current, we chose to cross the electrode wires in order to maximize the current through the brainstem. The brainstem contains the midbrain, pons, and medulla oblongata, where various complex nuclei control neurological functions such as the human cough and gag reflexes, and stimulation of the brainstem by CENA helps to strengthen the positive expression of neurons and the connection between the nuclei and the cerebral cortex, thus having a significant effect on the remodelling of the function of the patient's gag and cough reflexes. Stimulation of the brainstem by crossed electro-acupuncture helps to strengthen the positive expression of neurons and the connection between the nucleus pulposus and the cerebral cortex, so it has a significant effect on the remodelling of the patient's swallowing and coughing reflexes, and according to the results, the accompanying neurological recovery also helps the patient to pull out the tracheotomy cannula as soon as possible under the CENA treatment. Du (2012) found that the positive expression of Fos neurons was significantly increased by acupuncture at the TE17 and GB20 in SD rats, suggesting that stimulation of these two acupoints could directly or indirectly reach the dorsal cochlear nucleus (DCN), ventral cochlear nucleus thalamus (VCN), and inferior colliculus (IC), which in turn affected the electrical activity of the neural nuclei, that may verify our conjecture of therapeutic ideas [42]. In addition, the TE17 and GB20 acupuncture points are richly penetrated by blood vessels, such as the vertebral artery, the occipital artery, the lesser occipital nerve, and the inferior occipital nerve. Stimulation of these two acupuncture points can improve the blood supply to the basilar and internal carotid arteries and improve blood circulation to the cerebral cortex. The glossopharyngeal nerve, the vagus nerve, and the laryngeal nerve are fully nourished, thus restoring their functions.

Pseudobulbar palsy is usually treated clinically using a combination of Western and Chinese medicine. Western medicine is often used to activate blood circulation and promote nerve recoveries, such as cerebral protein hydrolysate tablets and olanzapine, which can gradually restore damaged nerves [43–45]. However, some adverse effects are often associated with Western medicine. Cerebral protein hydrolysate tablets may occasionally cause allergic reactions, including itching, rash, chills, low-grade fever, sometimes chest discomfort, headache, shortness of breath, and vomiting, and may trigger seizures and increase blood urea nitrogen [43, 44]. Olanzapine has led to psychotic excitement and sleep disturbances in a few patients, but nausea and gastric discomfort were only seen in a few patients in clinical trials, in addition to occasional pruritus, nausea, psychotic excitement, and sleep disturbances, but the symptoms were mild [45]. Therefore, it is clinically relevant to promote the use of CENA in the treatment of pseudobulbar palsy.

## 5. Conclusion

The clinical effects of CENA have been well established in this study, unfortunately, the validation at the neuronal level is lacking, which will be the next step in our research.

## Figures and Tables

**Figure 1:** Comparison of three groups of needling methods (a): Acupuncture group, (b): Electro-acupuncture group, and (c): CENA group.

**Figure 2:** Comparison of the three groups' scale scores after treatment: (a) Comparison of WST in the three groups after treatment; (b) Comparison of FDA in the three groups after treatment; (c) Comparison of TCRGS in the three groups after treatment; (d) Comparison of ChSWAL-QOL in the three groups after treatment.

**Figure 3:** The clinical efficacy comparison among three groups of patients (n).

**Table 1:** Acupuncture point selection.

Acupuncture point selection			
Shuigou (GV26);	Baihui (GV20);	Neiguan (PC6);	Dicang (ST4);
Jiache (ST6);	Lianquan (CV23);	Jinjin (EX-HN12);	Yuye (EX-HN13);
Jianyu (LI14);	Quchi (LI11);	Shousanli (LI10);	Huantiao (GB30);
Yanglingquan (GB33);	Jiexi (ST41);	Taichong (LR3);	Zusanli (ST36);
Sanyinjiao (SP6) act	Yifeng (TE17);	Fengchi (GB20)	

Acupuncture the contralateral motor area of the lesion (parietal temporal lobe anterior oblique line)			

**Table 2:** The water swallowing test (WST).

	The water swallowing test (WST)
Level I	Swallow the water once, <5 s, 30 ml water drunk, smoothly.
Level II	Swallow the water once or twice, >5 s, 30 ml water drunk, without choking cough.
Level III	Swallow the water once, 30 ml water drunk, with choking cough.
Level IV	Swallow the water over twice, 30 ml water drunk, with choking cough.
Level V	30 ml water drunk with difficulty, with many times of choking cough.

**Table 3:** Tracheostomy cough reflex grading score (TCRGS).

	Tracheostomy cough reflex grading score (TCRGS)
1 point	Patients with tracheotomy intubation persistently sealed time ≥24 hours, have a strong cough, and can spit out or swallow sputum spontaneously.
2 points	Patients with 12 h/d ≤tracheotomy intubation indirectly sealed time <24 h/d, with strong cough and partially spontaneous sputum, requiring passive aspiration of sputum ≤3 times/d.
3 points	Patients with tracheotomy intubation indirect sealed time <12 h/d, with strong cough and partially spontaneous sputum, requiring passive aspiration of sputum 4–6 times/d.
4 points	Patients with tracheotomy intubation incisions that cannot be sealed, coughing weakly, unable to sputum spontaneously, requiring passive aspiration of sputum 7–10 times/d, and shallow aspiration that induces a cough reflex.
5 points	Patients are unable to seal the tracheotomy intubation incisions, cough weakly, cannot spontaneously expel sputum, requiring passive aspiration of sputum >11 times/d, and deep coughing can induce cough reflex.

**Table 4:** Baseline data and characteristics ($\bar{x}$ ± *s*).

Item		CENA group	Electro-acupuncture group	Acupuncture group
Sample size (*n*)		40	40	40
Age (year)		55.87 ± 9.70	55.33 ± 10.11	55.88 ± 9.18
Gender (*n* (%))	Male	24 (60)	26 (65)	25 (62.5)
	Female	16 (40)	14 (35)	15 (37.5)
Course of the disease (d)		18.25 ± 3.73	18.68 ± 4.04	18.28 ± 3.73
Lesion location (*n* (%))	Cortex or subcortex	17 (42.5)	19 (47.5)	19 (47.5)
	Internal capsule or basal ganglia	23 (57.5)	21 (52.5)	21 (52.5)
Indexes before treatment *M (P*_*25,*_*P*_*75*_)	WST	4 (3, 5)	4 (3, 5)	4 (3, 5)
	FDA	10 (3.25, 14)	10 (4.25, 14)	11 (4.25, 15)
	TCRGS	4 (3, 4)	4 (3, 4)	4 (3, 4)
	ChSWAL-QOL	97 (87, 124.75)	99.5 (87, 124.75)	100 (87.25, 129)

*Note.* Age, gender, disease duration, and location of lesions were not statistically significant in the three groups, *p* > 0.05, and were comparable. SWT: No differences were found between the three groups (*h* = 0.7, *p*=0.75, *p* > 0.05); FDA: no differences were found between the three groups (*h* = 0.49, *p*=0.78, *p* > 0.05); TCRGS: no differences were found between the three groups (*h* = 0.047, *p*=0.977, *p* > 0.05); and ChSWAL-QOL: no differences were found between the three groups (*h* = 0.1.003, *p*=0.606, *p* > 0.05).

**Table 5:** The three groups of SWT, FDA, TCRGS, and ChSWAL-QOL levels were compared before and after treatment *M* (*P*_*25, *_*P*_*75*_).

Group	Time	WST (level)	FDA (item)	TCRGS (score)	ChSWAL-QOL (score)
CENA group	Before treatment	4 (3, 5)	10 (3.25, 14)	4 (3, 4)	97 (87, 124.75)
	After treatment	1 (1, 2)	26 (20, 27)	2 (1, 2)	150 (145, 170)
Electro-acupuncture group	Before treatment	4 (3, 5)	10 (4.25, 14)	4 (3, 4)	99.5 (87, 124.75)
	After treatment	2 (1, 3)^*∗*^	18.5 (15, 26)^*∗*^	2.5 (2, 3)^*∗*^	142.5 (127, 162.75)^*∗*^
Acupuncture group	Before treatment	4 (3, 5)	11 (4.25, 15)	4 (3, 4)	100 (87.25, 129)
	After treatment	3 (2, 4)^*∗*^#	16 (10, 19)^*∗*^#	3 (2, 4)^*∗*^#	128.5 (112.25, 148.75)^*∗*^#

*Note.* ^*∗*^ *P* < 0.001, after treatment, compared with the CENA group; #*P* < 0.001, after treatment, compared with the electro-acupuncture group.

**Table 6:** The clinical efficacy comparison among three groups of patients (n (%)).

Group	Sample size (*n*)	Cure	Significant effect	Effective	Ineffective
CENA group	*n* = 40	21 (52.5)	14 (35.0)	3 (7.50)	2 (5.0)
Electro-acupuncture group	*n* = 40	12 (30.0)	8 (20.0)	14 (35.0)	6 (15.0)
Acupuncture group	*n* = 40	3 (7.5)	5 (12.5)	18 (45.0)	14 (35.0)
*X* ^*2*^			38.7		
*p*			*p* < 0.001		

## Data Availability

All data generated or analysed during this study are included in this published article.
